The article "Mesenchymal Stem Cell Therapy: A Potential Treatment Targeting Pathological Manifestations of Traumatic Brain Injury" was published in 2022. Journal: Oxid Med Cell Longev.

# Mesenchymal Stem Cell Therapy: A Potential Treatment Targeting Pathological Manifestations of Traumatic Brain Injury

**DOI:** 10.1155/2022/4645021

**Published:** 2022-06-15

**Authors:** Kaige Zhang, Yiming Jiang, Biyao Wang, Tiange Li, Dehao Shang, Xinwen Zhang

**Affiliations:** ^1^Center of Implant Dentistry, School and Hospital of Stomatology, China Medical University, Liaoning Provincial Key Laboratory of Oral Diseases, Shenyang, China; ^2^The VIP Department, School and Hospital of Stomatology, China Medical University, Liaoning Provincial Key Laboratory of Oral Diseases, Shenyang, China

## Abstract

Traumatic brain injury (TBI) makes up a large proportion of acute brain injuries and is a major cause of disability globally. Its complicated etiology and pathogenesis mainly include primary injury and secondary injury over time, which can cause cognitive deficits, physical disabilities, mood changes, and impaired verbal communication. Recently, mesenchymal stromal cell- (MSC-) based therapy has shown significant therapeutic potential to target TBI-induced pathological processes, such as oxidative stress, neuroinflammation, apoptosis, and mitochondrial dysfunction. In this review, we discuss the main pathological processes of TBI and summarize the underlying mechanisms of MSC-based TBI treatment. We also discuss research progress in the field of MSC therapy in TBI as well as major shortcomings and the great potential shown.

## 1. Introduction

More than 50 million people worldwide suffer from traumatic brain injury (TBI) annually, creating a significant burden on society and families [1]. It has also been shown that TBI is associated with an increased incidence of common neurodegenerative diseases such as Alzheimer's disease (AD) [2, 3] and Parkinson's disease [4, 5]. Severe TBI can trigger a long-term neurodegenerative process leading to pathological features and clinical manifestations similar to those of neurodegenerative diseases such as AD, structural destruction of neurons and functional impairment, and memory and cognitive decline, which in turn affect speech and motor systems [6]. TBI refers to the physical damage to brain tissue caused by a violent blow to the head. The primary injury results from direct mechanical injury. The secondary injury is characterized by diffuse axonal injury and inflammation that can protect tissues from pathogens and remove cell debris; however, severe cases can lead to neurodegeneration and secondary neuron death [7–9]. The secondary injury is a progressive process that lasts from hours to days, which means that therapeutic interventions can be administered at this stage to avoid progressive nerve cell death and enhance functional recovery after brain trauma. TBI may disrupt the blood–brain barrier (BBB) to cause neurochemical, metabolic, and cellular changes [10–12] and activate microglia and astrocytes.

The activation of microglia and astrocytes leads to the removal of cellular debris, restoration of the BBB, and production of neurotrophic factors [13]. However, inflammatory cells, such as neutrophils, are recruited to accelerate the inflammatory response and cause damage to peripheral tissues [14, 15]. The adult brain undergoes limited remodeling to compensate for tissue damage after TBI [16]. Therefore, new treatments for TBI can be developed by elucidating brain tissue remodeling and internal repair processes.

Over the past few decades, treatment for TBI has always been a focus of attention. Three main options are commonly used to treat TBI: hypothermic therapies reduce intracranial pressure, decrease inflammatory responses, and lower cerebral metabolic rate [17]. Surgical therapies remove most of the skull bone by debridement decompression to reduce intracranial pressure and remove hematomas [18]. Pharmacological therapies reduce active bleeding, nourish the nerves, are anti-inflammatory, and include erythropoietin [19], tranexamic acid [20], and recombinant interleukin-1 receptor antagonist [21, 22].

The latest studies have shown that mesenchymal stromal cells (MSCs) have great potential in treating TBIs due to their anti-inflammatory and antiapoptotic properties and the ability to generate new nerves. Similarly, extracellular vesicles (EVs) released by MSCs cross the BBB and promote endogenous angiogenesis and neurogenesis, reduce inflammation, and facilitate cognitive and sensorimotor recovery after TBI. Taken together, this suggests that MSCs may be a promising cell-free therapy for TBI [23]. In this review, we summarize the possible molecular or cellular mechanisms of MSCs as a therapeutic approach in TBI pathology. At the same time, the prospect of cellular therapy, represented by MSCs and exosome-based, cell-free therapy, is analyzed to demonstrate its therapeutic potential.

## 2. TBI-Based Functional Features of MSCs

To date, 125 clinical trials have been conducted using MSCs for neurological diseases [24], including TBI treatment. The administration of autologous bone marrow MSCs (BM–MSCs) to patients during the subacute phase of TBI resulted in improved neurological function in 40% of patients [25]. A stem cell is a type of cell that is not highly differentiated and has the potential to regenerate various tissues, organs, and the human body. These cells can be classified into totipotent stem cells, multipotent stem cells, and unipotent stem cells according to different differentiation potentials. Stem cells can be induced to proliferate and differentiate into corresponding tissues and organs under appropriate conditions, which is of extraordinary significance in clinical treatment. MSCs are multipotent stem cells with self-renewal and multidifferentiation abilities [26]. These cells are widely found in a variety of tissues throughout the body and can be isolated from many sources, including BM [27], synovial membrane, skeletal muscle [28], adipose tissue [29], and peripheral blood [30]. MSCs can differentiate into mesodermal cells and tissues in different microenvironments [31]. Such cells have the advantages of easy access, low immunogenicity, regenerative potential even after freezing, and the ability to migrate to the lesion [32]. These characteristics make MSCs a promising regenerative treatment for brain trauma. Initially, the therapeutic efficacy of MSCs was thought to be based on their ability to differentiate and replace damaged cells. However, recent studies have revealed that the repair of damaged tissues is mainly through cell–cell interactions, paracrine effects, and the release of EVs [33, 34]. In a rat model of TBI, intravenously administered BM-MSCs can penetrate the BBB and increase trophic factors in the brain [35]. They can also selectively migrate to injured areas of brain tissue and differentiate into neurons and astrocytes [36]. Promoting axonal remodeling in the brain and angiogenesis and glial cell growth at the site of injury can accelerate the internal repair process while achieving the goal of promoting neuroprotection, neurorepair, and restoration of motor function.

Exosomes are small vesicles with a 50-200 nm diameter containing RNA, mRNA, DNA, and biologically active substances such as proteins and lipids [37]. Released from numerous cells, exosomes play a key role in intercellular signal transduction in physiological or pathological processes [38]. BM-MSC-derived exosomes reduce neuroinflammation by releasing anti-inflammatory cytokines and affecting the apoptosis of activated T cells [39, 40]. It was found that MSCs promoted neurological recovery in a rat model of TBI [41]. Even the exosomes secreted by MSCs under hypoxic conditions can delay neuronal degeneration and promote neural recovery [42]. Studies have shown that EVs have low immunogenicity and the ability to stimulate neurovascular repair, characteristics similar to those of MSCs. Compared to MSCs, EVs are more stable and equally capable of crossing the BBB. The use of EVs reduces safety issues associated with the administration of live cells, such as microvascular obstruction and abnormal growth of transplanted cells [43]. In addition, they have the advantages of being free of ethical problems, are less invasive, and show low tumorigenicity [44], which has extraordinary significance for their wide range of applications. The cell source of exosomes can be clonally selected to ensure their standardization and reproducibility, making the industrial production of exosomes more promising [45]. However, proteomic analysis revealed differences between human MSC-derived exosomes isolated from BM, adipose, and human umbilical cord perivascular cells [46]. More studies are therefore needed to determine the best choice of MSCs for exosomes to be used in TBI treatment.

In short, MSCs and their secreted exosomes are promising candidates for TBI treatment. Many clinical studies are underway to determine the optimal route and time of administration and dosage of MSCs and exosomes, which are popular directions for future research.

## 3. The Role of MSCs in Treating TBI

### 3.1. Mitochondrial Dysfunction and Transfer

Mitochondria not only produce adenosine triphosphate (ATP) for various metabolic activities but are also involved in regulating cell death. In TBI-related neurological injury, secondary injury is mainly caused by mitochondrial dysfunction [47]. Damaged mitochondria trigger a chain of pathological events [48], such as excitotoxicity, increased reactive oxygen species (ROS) production, oxidative stress, mitochondrial DNA damage, and mitophagy [49], leading to decreased cellular energy production [47] and apoptosis. Due to the prevalence of mitochondrial dysfunction in TBI, one potential therapeutic target is to improve mitochondrial function. Numerous studies have focused on mitochondria as therapeutic targets for acute brain injury in recent years. For example, therapies that reverse mitochondrial uncoupling, increase mitochondrial antioxidant production, or inhibit mitochondrial permeability transition pores (MPTP) have been investigated [50]. Neuroprotective therapies have also been identified as promising therapies. Reperfusion strategies, hemoglobin management, and therapeutic (induced) hypothermia do well in neuroprotective therapy [51]. As a new mechanism of stem cell therapy, MSC-derived mitochondrial transplantation has achieved promising results [52]. A series of preclinical studies and clinical trials have shown that MSCs can transfer mitochondria to damaged cells via various routes [34], replace defective mitochondria, or compensate for their dysfunction [53]. Mitochondrial transfer protects cells from damage and apoptosis by increasing mitochondrial membrane potential, restoring aerobic respiration, or reducing inflammation. As previously mentioned, neurogenic inflammation is a pathological manifestation of TBI [52]. Studies have shown that MSCs moderate secondary injury due to inflammation [54]. Mitochondria can be transferred between MSCs and immune cells, including macrophages and T cells [55], regulating their functions and changing cytokine expression profiles. Morrison et al. reported that MSCs could donate mitochondria to host macrophages, leading to suppressed cytokine production, increasing M2 macrophage marker expression, and enhanced macrophage phagocytosis [56].

Furthermore, in rats, transferred mitochondria have been shown to enhance angiogenesis and improve functional recovery of the brain microvascular system [57]. In the process of neuronal apoptosis involved in mitochondria, B-cell lymphoma 2 (Bcl-2) family proteins are proapoptotic factors and promote mitochondrial membrane permeability [58]. An apoptotic cascade is triggered, and caspases (including caspase-3) are activated, resulting in caspase-dependent DNase proteolysis and internucleosomal DNA fragmentation [59]. Mitochondrial transfer from MSCs can decrease apoptosis rates in recipient cells and improve cell survival [60] by regulating the Bcl-2-associated X protein (Bax)/Bcl-2 ratio and decreasing caspase-3 expression [61]. The protective effect of mitochondrial transfer therapy on nerves and the restoration of spinal cord function are apparent. Research has indicated that mesenchymal multipotent stromal cells can supply mitochondria to damaged astrocytes [62]. The transfer of MSC-derived mitochondria to oxidant-damaged neurons may help increase neuronal survival and improve metabolism [63]. In a spinal cord injury rat model, mitochondria can be transferred from BM-MSCs to injured motor neurons to significantly improve locomotor functions six weeks after injury [64].

A growing body of research suggests that intercellular mitochondrial transfer between MSCs and target cells occurs through tunneling nanotubes (TNTs) [65], microvesicles [66], EVs, gap junctions, and cytoplasmic fusion [67, 68]. At present, the formation of TNTs is the most widely accepted theory. TNTs are a type of nanotube that can transport substances directly between cells, including proteins, ions, RNA, organelles, viruses, and cytosol [69]. Thus, although mitochondrial transfer is directed and mostly one-way transportation [52], it can also manifest as bidirectional transportation [70], meaning that MSCs may exchange mitochondria with other types of cells. The regulation of mitochondrial transport directionality remains to be studied further. Mitochondria also play a regulatory role in the renewal and differentiation of MSCs. In other words, a bidirectional interaction exists between mitochondria and MSCs.

In addition, mitochondrial transfer therapy has other potential dangers. Transferred mitochondria support tumor progression by providing energy to cancer cells [71] and increasing drug resistance [72]. A tumor-induced inflammatory response leads to the production of chemokines, which attract MSCs to the site of inflammation. Due to good differentiation capabilities, MSCs can differentiate into cancer-induced fibroblasts. Such fibroblasts play a role in immune regulation thus promoting the growth and migration of cancer cells. Studies have shown that MSCs can transport mitochondria to breast cancer cells and glioblastoma stem cells to promote tumor growth. Studies have found that MSCs transfer cytoplasmic content but not mitochondria to cancer cells and may lead to chemotherapy resistance in cancer cells. However, the specific mechanism of mitochondrial transport between MSCs and other cells is still unclear. Therefore, in some cases, mitochondrial transfer should be suppressed. It is worth mentioning that the source and status of MSCs also affect mitochondrial transfer. The mitochondrial transferability of MSCs isolated from different tissue sources varies. The therapeutic effects of damaged or aged MSCs are limited and unsuitable for stem cell therapy. In inflammatory environments, the formation of TNTs is inhibited, thus affecting the transport of mitochondria from MSCs to damaged cells. Therefore, the MSC source should also be considered.

### 3.2. Oxidative Stress

Oxidative stress is a disorder in the generation and removal of ROS, a double-edged sword. While causing some damage, ROS also stimulate repair. When excess radicals are produced, repair processes are impaired, leading to oxidative stress and cell death through apoptosis or necrosis [73]. Studies have shown that during secondary TBI injury [74], free radical production and oxidative damage are influential in neuronal structures (e.g., axons). After axon injury, excessive Ca^2+^ influx can cause mitochondrial dysfunction and ROS overproduction [75]. ROS can destroy the integrity of cell membranes and cause cell damage through lipid peroxidation, protein, and DNA oxidation and the inhibition of mitochondrial electron transport chains. ROS can also activate microglia in the brain to release inducible nitric oxide synthase (iNOS) and cytokines, leading to inflammation and cell death [76].

Meanwhile, due to a lack of introns and its proximity to the source of ROS, mitochondrial DNA (mtDNA) is liable to oxidative damage. This may lead to decreased respiratory function and promote ROS production—a vicious cycle that eventually induces apoptosis [77]. ROS are also known to trigger the mitochondrial apoptosis cascade through interaction with the permeability transition pore complex protein [78]. The importance of oxidative stress in mitochondrial dysfunction and neuronal death after acute brain injury cannot be ignored and suggests that targeted therapy is promising.

Many studies have shown that MSCs can protect brain tissue from severe damage by inhibiting oxidative stress. In a TBI mouse model, overexpression of specific genes, such as that for superoxide dismutase 2, *in vitro* can enhance the antioxidant effect of MSCs and improve their therapeutic effect [79]. Histone deacetylase 1 (HDAC1) promotes stromal cell self-renewal and disease recovery by enhancing histone acetylation [80]. Silencing HDAC1 in MSCs attenuates oxidative stress and neuroinflammation, thus improving its therapeutic effect [81]. *In vitro* studies have found that mitochondria from MSCs are reduced in mouse neurons following hydrogen peroxide exposure [63]. Transferring mitochondria from MSCs to neurons impaired by oxidative stress may contribute to the preservation of posttraumatic neurons and restore their function. In addition, it has been shown that MSCs can mitigate the effects of oxidative stress in the central nervous system by changing the activity of ascorbic acid and catalase [82]. MSCs can also increase expression of the antiapoptotic gene, *Bcl-2*, and decrease the level of superoxide anion, thereby protecting brain tissue [83]. Olfactory mucosa MSCs are helpful in antioxidative stress and neuroprotection by upregulating *SPCA1* expression, reducing Ca^2+^ overload and Golgi edema and lysis, therefore, playing a significant role in combatting oxidative stress and facilitating neuroprotection [84]. In addition, exosomes produced by MSCs can increase ATP production, reduce oxidative stress, and activate the phosphoinositide 3-kinase/Akt pathway [85], which is of great value for the application of exosomes in TBI treatment. MSC-derived EVs inhibit proinflammatory responses and reduce oxidative stress and fibrosis in *in vivo* models [86]. The above results show that MSCs play a significant role as antioxidants in treating TBIs.

In addition, during oxidative stress, astrocyte-derived exosomes transport neuroprotective apolipoprotein D to neurons to improve the neuronal survival rate [87]. Meanwhile, astrocyte-derived exosomes protect hippocampal neurons after TBI by activating the nuclear factor erythroid 2-related factor 2 signaling pathway in animal models to prevent TBI-induced oxidative stress and neuronal apoptosis [88]. Recent studies have shown that micro (mi)RNAs within astrocyte exosomes are different under proinflammatory and oxidative stress conditions versus the resting state [89]. This has important implications for future studies on the potential role of miRNAs in cellular communication, inflammation, and exosome therapy for TBI.

### 3.3. Neuroinflammation

Neuroinflammation is associated with secondary TBI injury [90]. TBI leads to neuronal damage and damages the integrity of the BBB. Immune cells invade and activate glial cells such as microglia and astrocytes [91, 92]. Microglia polarize to the M1 (proinflammatory) phenotype, and expression of the surface protein cluster of differentiation 14 (CD14) is promoted, which is a sign of acute inflammation caused by TBI. Glial cells continuously release inflammatory mediators, such as interleukin- (IL-) 1, IL-6, tumor necrosis factor- (TNF-) *α*, and other cytokines, to attract more peripheral macrophages and neutrophils across the leaky BBB, consequently converting inflammation from the acute to chronic phase [93]. At the same time, neurons and microglia are damaged, and cellular adhesion molecules and matrix metalloproteinases are secreted in addition to immune cells. The persistent TBI-induced inflammation can result in neuronal loss and cerebral edema [94] and lead to degenerative diseases such as AD [95]. TBI can also cause peripheral inflammation, mainly in the spleen and thymus, which may lead to multiple organ dysfunction and even death. Studies have shown that plasma levels of inflammatory molecules begin to rise 6 hours after TBI and continue to increase [96]. The release of these inflammatory molecules, including TNF-*α*, IL-6, and ROS, promotes systemic diseases such as cancer, atherosclerosis, and diabetes. Neuroprotective and anti-inflammatory drugs are potential therapies for TBI. Many preclinical studies and clinical trials have demonstrated that MSCs can regulate the inflammatory microenvironment, thus decreasing inflammation and immune reactions to promote tissue repair [97, 98]. The therapeutic effects of MSCs regarding neuroinflammation are achieved through paracrine factors [99]. Following implantation, MSCs cross the BBB, migrate to the site of injury, and release trophic factors to recover neuronal structure and function [100]. MSCs regulate innate and adaptive immune cells by releasing soluble factors to enhance anti-inflammatory pathways at the site of injury [101]. A study in a TBI rat model showed that MSCs decreased the number of microglia and other inflammatory cells, reduced the production of proinflammatory cytokines, and increased anti-inflammatory cytokines to inhibit TBI-induced inflammatory responses. MSCs enhance TNF-stimulated gene 6 expression, which suppresses the NF-*κ*B signaling pathway [102]. When BM-MSCs were administered seven days after TBI, a 50% reduction in interferon-*γ* and TNF-*α* expression was observed, as well as an increase in neurogenesis and a significant decrease in BBB permeability, edema, microglial activation, and norepinephrine levels [103, 104]. A recent study of 20 patients with severe TBI showed that after successful intravenous MSC treatment, the percentage of neutrophils in the blood decreased significantly to normal levels, and the production of IL-6, C-reactive protein, TNF-*α*, and ROS also decreased. It is suggested that MSC therapy restricts the accumulation of immune cells and systemic inflammatory cytokines at the injured site. In addition, compared with the control group, the Glasgow score and Health Stroke Scale of the group treated with MSCs increased starting on the seventh day post-TBI. This proved that MSC therapy contributed to the recovery of motor function and consciousness in patients with TBI [96].

Moreover, MSCs inhibit phagocytosis and stimulate microglial polarization to the more neuroprotective and anti-inflammatory M2 phenotype, thereby ameliorating functional deficits in rats with TBI [105]. Studies have shown that proteins in BM-MSC-exosomes injected into C57BL/6 male mice can downregulate iNOS and upregulate CD206 and arginase-1, resulting in polarization of microglia/macrophages and inhibition of early neuroinflammation in TBI [106]. MSCs can also suppress T cell proliferation and monocyte differentiation, thus affecting dendritic cell functions and increasing the production of IL-10 [100].

Many studies have shown that infusion is a common method of drug administration in stem cell therapy. Intranasal secretome administration has been assessed as a noninvasive and efficient route of administration that targets cells to the brain [107]. Administering autologous BM–MSCs by lumbar puncture has also been shown to be a safe and efficient cell therapy [25]. Focal intracerebral transmission of MSCs may be more suitable for focal injury as this will directly target areas of inflammation [105]. Compared to monotherapy, combination therapy that includes regulatory T cells and MSCs enhances potency and significantly attenuates inflammation after TBI [108]. Combined BM-MSCs and the peroxisome proliferator-activated receptor gamma agonist, pioglitazone [109] or propranolol [103] can also enhance anti-inflammatory effects. Several studies have shown that intravenous injection of BM mononuclear cells followed by MSCs improves cognitive function in patients with TBI [96]. A few studies showed that the reaction of host immune cells to the transplanted MSCs may be harmful [110]. Therefore, more research is needed to understand the long-term impact of stem cell therapy.

### 3.4. Apoptosis

In addition to trauma-induced primary damage to the BBB and neuronal death, neuronal and oligodendrocytic apoptosis is a marker of secondary brain injury [111]. After TBI, significant nerve cell death can be found in the hippocampus. The cell fragments released from the damaged site can activate an immune response from microglia and astrocytes, resulting in the release of inflammatory factors and result in neuroinflammation. The release of TNF-*α* can activate the caspase-3 signaling pathway and induce neuronal apoptosis. Neuronal apoptosis is dependent on the opening of MPTP and the release of cytochrome C [50, 112]. Cytochrome C forms an apoptosome in the cytosol by interacting with the protein cofactor, apoptotic protease activating factor-1, to trigger an apoptotic cascade. The complex activates procaspase-9 and induces a caspase-9-dependent intrinsic pathway [113]. Subsequently, caspase-3 and other caspases are activated resulting in caspase-dependent DNase proteolysis and internucleosomal DNA fragmentation [59]. Mitochondrial pathway-induced apoptosis can be ameliorated by mitochondrial transfer of MSCs. The paracrine mechanism of MSCs promotes angiogenesis and is anti-inflammatory and antiapoptotic [114]. Many studies have shown that MSCs can improve neuronal survival and cure brain injury by interfering with the apoptotic pathway [100]. An experiment by Mettang et al. found elevated levels of the proapoptotic mediators, Bax and Bad, in a closed head injury model of TBI [115]. A recent study showed that the neurological function of C57BL/6 male mice treated with 30 *μ*g protein equivalent of BM-MSC-exosomes was significantly improved compared to control mice. The expression of the proapoptotic protein, Bax, was inhibited, while the expression of the antiapoptotic protein, Bcl-2, was enhanced. Injection of MSC-EVs into 3-day-old Wistar rats decreased nerve cell death, white matter microstructure destruction, and glial cell proliferation induced by lipopolysaccharides [116]. MSCs can also downregulate caspase-3, promote the production of antioxidants, and secrete neurotrophic factors such as neurotrophin-3 [117]. In addition, various nutritional factors secreted by MSCs can inhibit endothelial cell apoptosis [118] and promote the formation of new capillary branches in injured brain tissue [119]. Angiogenic paracrine factors of MSCs include human vascular endothelial growth factor, transforming growth factor-*β*1, monocyte chemotactic protein-1, and IL-6 [120]. These factors have been proved to reduce apoptosis and injury volume and improve motor and cognitive impairment in patients. The paracrine effects of MSCs play an essential role in regulating apoptosis pathways, thereby improving neuronal survival rate, promoting angiogenesis, repairing nerve injury, and maintaining the physiological functions of the brain.

## 4. Comparison of Existing Therapies

With its severe and complex secondary pathologies, TBI has greatly affected patients' quality of life and brought a medical burden onto their families and society. In the past few decades, traditional treatments, such as hypothermic therapies, surgery, and drug therapies, have been the main treatments for TBI. Medical interventions, such as drug and hypothermia therapies, are usually considered for patients with mild to moderate TBI. Invasive surgical treatment is needed for extra-axial hematoma, concussions, and brain edema. However, limitations exist with traditional treatments. Specifically, the focus is on the relief of physiological symptoms to maintain quality of life. However, treatment efficacy is limited and is more likely to cause secondary trauma. In addition, the pain of long-term sequelae and lifelong disability cannot be prevented. In recent years, stem cell therapy has become more popular. Stem cell transplantation can prevent or reverse damage at the biochemical and cellular levels and relies on endogenous healing mechanisms to restore brain function. For elderly patients with TBI, a combination of cell transplantation and other treatments, such as cooling and electrical stimulation, may be needed to promote brain repair. Stem cell therapy may be more effective in promoting neuronal regeneration in young people [121]. Stem cells can be divided into hematopoietic stem cells, MSCs, neural stem cells (NSCs), epithelial stem cells, and skin stem cells. Recent studies have shown that various stem cells can treat neural damage after TBI, including MSCs, NSCs, multipotent adult progenitor cells, and endothelial progenitor cells. Of these, MSCs have the most significant therapeutic potential because of the ease of isolation, low immunogenicity, and ability to differentiate into various tissue lineages, including brain cells [122]. However, several limitations still exist for MSC transplantation. Contamination is probable during the culture and treatment of MSCs, and *in vitro* cultured cells are prone to mutation. Cell transplantation may also lead to the transmission of foreign pathogens. In addition, MSC transplantation may provide energy for cancer cells and promote tumor growth and metastasis. The initiation and regulation of mitochondrial transfer from MSCs are not clear. Additionally, the probability of allogeneic immune rejection cannot be ignored. Therefore, it is particularly important to improve the safety of MSC therapy.

## 5. Conclusion and Future Perspectives

The treatment of TBI has received much attention due to its high morbidity and complex secondary cascades. Oxidative stress, neuroinflammation, neuronal apoptosis, and mitochondrial dysfunction are all classic pathological manifestations of TBI. In recent years, MSC transplantation has been investigated as a therapeutic approach due to its ability to repair damaged brain tissue in TBI models. Transplanted MSCs can pass through the BBB and migrate to damaged brain tissue to play a therapeutic role through multidirectional differentiation, paracrine effects, and the release of EVs. Apart from secreting nutritional factors to exert anti-inflammatory effects and promote angiogenesis, MSCs can also transfer mitochondria to damaged neurons via TNTs (Figure 1). Compared with traditional therapies, MSC treatment can directly improve TBI-induced pathological changes and promote recovery of neurological function. However, the efficacy and safety of MSCs as a potential therapy for TBI remain controversial. Available preclinical studies have shown that the excellent repairability of MSC may sometimes be translated into oncogenic ability. The potential risk of an immune response by the host's own immune cells to MSCs is unclear. In addition, the appropriate timing of drug administration, more efficient routes of administration, reliable cell sources, and methods of cell culture, storage, and transportation are all worthy of discussion. Insufficient clinical trials have been conducted to demonstrate a direct therapeutic effect of MSC therapy on the pathological manifestations of TBI. In a series of clinical studies on stroke, despite the fact that MSCs isolated from different tissues were effective in treating this disease, disparities in efficacy existed between trials. Although transporting MSCs through the intracerebral pathway is most effective, it is also the most invasive. In contrast, the intravenous route is the least invasive and reaches the least number of MSCs in the damaged brain tissue. Therefore, it may be challenging to obtain stable cells, deliver MSCs accurately through a safe delivery method, and obtain stable efficacy of MSC therapy for TBI. MSC therapy can be optimized in several ways. For example, genetically modified MSCs can be the basis for the next generation of cell-based therapies for TBI. In addition, compared to monotherapy, combination therapy with other drugs can enhance the effectiveness of treatment. Furthermore, the use of MSC-derived exosomes can avoid several problems associated with cell transplantation. However, further preclinical and clinical studies are needed to discover the therapeutic potential of MSCs.

## Figures and Tables

**Figure 1:** TBI pathology and MSC-related treatment mechanisms. When TBI occurs, the BBB is disrupted, leading to a series of responses such as hypoxia, edema, and release of inflammatory factors by immune cells. Excessive production of ROS in neurons and alteration of mitochondrial membrane potential results in a variety of pathological processes, such as oxidative stress, mtDNA damage, mitophagy, and apoptosis, some of which will eventually lead to cell death. Furthermore, they also enable MPTP to open instantly promoting the above pathological processes. When we use MSCs to treat TBI, MSCs and their released exosomes can cross the BBB stably and release various cytokines, such as neurotrophic factors and vascular regeneration factors, to promote nerve and blood vessel repair and regeneration. MSCs can also deliver healthy mitochondria to neurons through TNTs to enhance the anti-inflammatory, antioxidant, and antiapoptotic abilities of neurons and eventually improve their functions. BBB: blood-brain barrier; MSC: mesenchymal stromal cell; MPTP: mitochondrial permeability transition pores; mtDNA: mitochondrial DNA; ROS: reactive oxygen species; TBI: traumatic brain injury; TNT: tunneling nanotubes.
